The article "PyraPVConv: Efficient 3D Point Cloud Perception with Pyramid Voxel Convolution and Sharable Attention" was published in 2022. Journal: Comput Intell Neurosci.

# PyraPVConv: Efficient 3D Point Cloud Perception with Pyramid Voxel Convolution and Sharable Attention

**DOI:** 10.1155/2022/2286818

**Published:** 2022-05-13

**Authors:** Yuhong Chen, Weilong Peng, Keke Tang, Asad Khan, Guodong Wei, Meie Fang

**Affiliations:** ^1^Guangzhou University, Guangzhou, China; ^2^South China University of Technology, Guangzhou, China

## Abstract

Designing efficient deep learning models for 3D point cloud perception is becoming a major research direction. Point-voxel convolution (PVConv) Liu et al. (2019) is a pioneering research work in this topic. However, since with quite a few layers of simple 3D convolutions and linear point-voxel feature fusion operations, it still has considerable room for improvement in performance. In this paper, we propose a novel pyramid point-voxel convolution (PyraPVConv) block with two key structural modifications to address the above issues. First, PyraPVConv uses a voxel pyramid module to fully extract voxel features in the manner of feature pyramid, such that sufficient voxel features can be obtained efficiently. Second, a sharable attention module is utilized to capture compatible features between multi-scale voxels in pyramid and point cloud for aggregation, as well as to reduce the complexity via structure sharing. Extensive results on three point cloud perception tasks, i.e., indoor scene segmentation, object part segmentation and 3D object detection, validate that the networks constructed by stacking PyraPVConv blocks are efficient in terms of both GPU memory consumption and computational complexity, and are superior to the state-of-the-art methods.

## 1. Introduction

With the advance of depth sensing devices, 3D point clouds can be captured in a much easier manner. Therefore, applications of 3D point cloud perception are now booming, e.g., simultaneous localization and mapping (SLAM) [1–3], and autonomous driving [4–6]. In the last few decades, 3D point cloud perception mainly depends on hand-crafted shape descriptors [7–9]. Until very recently, researchers start to extend deep learning models which are mature in the field of 2D computer vision to handle 3D perception tasks, significantly refreshing the state-of-the-art records [10–12]. However, 3D deep learning models with higher accuracies always have higher complexities, which now becomes the major obstacle for their application to real-world scenarios.

There have been many attempts that utilize deep networks to perceive 3D point clouds. According to the representation of data that feeds to deep networks, these methods could be divided into two categories broadly: structure-based methods and point-based methods. Structure-based methods first convert irregular point clouds into structured grid representations, e.g., projecting point clouds into bird's eye views [13, 14] or rasterizing into 3D voxel grids [10, 15–17], and then adopt traditional 2D convolutional neural networks (CNNs) or their simple extensions to extract discriminative CNN features. However, it introduces exponential computational cost and memory for detailed 3D geometric learning at high resolutions. Point-based methods instead impose multi-layer perceptrons (MLPs) followed with maximum pooling [11, 18] or irregular kernels [19] to 3D point clouds, such that they can handle points directly. Nevertheless, since these methods require accessing irregularly scattered points especially for local feature aggregation, they are also inefficient.

The article "PyraPVConv: Efficient 3D Point Cloud Perception with Pyramid Voxel Convolution and Sharable Attention" was published in 2022. Journal: Comput Intell Neurosci.

By analysing both the advantages and disadvantages of structure-based and point-based methods, the pioneering point-voxel convolution (PVConv) [20] proposes to combine them together for efficiency purpose. Particularly, point-based MLPs are adopted to extract 3D features in the point branch; and voxel convolutions aggregate local features coarsely in the voxel branch; in addition, linear interpolation is conducted to fuse the features of the two branches. PVConv brings large improvements in terms of GPU memory consumption and computational efficiency, but the accuracy of PVConv is somewhat sacrificed. By going through the structure of PVConv, we hypothesize that there are two key factors that limit its performance. First, the voxel-based networks with strong feature extraction capabilities are utilized too conservatively, i.e., with only two layers of simple 3D convolutions. Second, the voxel features that are already insufficient would further lose during the fusion process, since it is implemented via a linear-based interpolation that is not powerful enough.

To resolve the above two issues, we intentionally design a novel pyramid point-voxel convolution (PyraPVConv) block. First, we adopt a more powerful 3D voxel convolution branch that extracts multi-scale voxel features in the form of feature pyramid, such that powerful 3D voxel convolutions can be fully exploited with sacrificing moderate additional computational overhead. Second, to alleviate the information loss during the feature fusion process between point and voxel branches, we propose utilizing the attention mechanism to learn to combine them in a more compatible way. Particularly, we design a sharable attention module that learns the relevant scores between multiple voxel branches and the point branch with sharing a structure, such that it reduces the overhead required by multibranch attention. With these two designs against the weaknesses of PVConv, the PyraPVConv block can perceive 3D point clouds in a better tradeoff between accuracy and efficiency.

The article "PyraPVConv: Efficient 3D Point Cloud Perception with Pyramid Voxel Convolution and Sharable Attention" was published in 2022. Journal: Comput Intell Neurosci.

Overall, our contribution is three-fold.

- We propose a lightweight 3D perception block, PyraPVConv, that can perform 3D point cloud perception accurately and efficiently
- We design a voxel pyramid module, which better extracts voxel features without introducing too much additional computational overhead
- We devise a sharable attention module that fuses the features of point branch and multiple voxel branches in a more effective nonlinear manner

We construct PyraPVCNN by stacking multiple PyraPVConv blocks following PVCNN [20], and evaluate it on various point cloud perception tasks, e.g., indoor scene and object part segmentation, 3D object detection. Extensive experiments demonstrate the superiority of PyraPVConv to the state-of-the-art methods in terms of both accuracy and efficiency.

## 2. Related Work

### 2.1. Efficient Deep Learning for Point Clouds

Deep learning techniques have been widely adopted for handling 3D point cloud perception tasks, e.g., classification and segmentation, by projecting sparse point clouds into compact semantic representations [21–25]. However, as indicated in [20], most current 3D deep learning methods for point clouds are less efficient, e.g., voxel-based methods require large amounts of memory for maintaining detailed 3D structures, and point-based methods require high CPU latency to search neighborhood points for feature aggregation.

To perceive 3D point clouds in a more efficient way, Liu et al. [20] proposed the point-voxel convolution (PVConv), that combines point-based MLPs for individual point feature extraction and voxel-based CNNs for neighborhood feature aggregation. Since with only two layers of simple 3D CNNs, the performance of PVConv is somewhat sacrificed. To better utilize the voxel information, Tang et al. [26] further designed sparse point-voxel convolution (SPVConv), which uses sparse convolution to handle high-resolution voxels on the basis of PVConv, and further adopted network architecture search (NAS) for searching the best architecture. Although their method showed good performance in large-scale scenarios, sparse convolution is complex and is less efficient in common scenes. Our method also aims to fully utilize 3D voxel information. Differently, we adopt the concept of feature pyramid to balance the accuracy and efficiency.

We also notice some other works that also aim to efficient point cloud learning by randomly key point sampling [27], by irregularly volume partition [28], and by leveraging mature 2D methods [29], etc., but these directions are out of our scope.

The article "PyraPVConv: Efficient 3D Point Cloud Perception with Pyramid Voxel Convolution and Sharable Attention" was published in 2022. Journal: Comput Intell Neurosci.

### 2.2. Multiscale Feature Modeling

Modeling multi-scale features has been validated to be a useful strategy in computer vision, e.g., maintaining scale-invariant property in SIFT [30] and controlling the receptive field in CNNs [31]. This strategy is also widely adopted in 3D deep learning. PointNet++ [18] extracts multi-scale features of point clouds by hierarchically applying PointNets [11]. 3D object detection frameworks [17, 32, 33] adopt different detection heads with multi-scale feature maps to handle both large and small object classes. ContFuse [34] uses continuous convolution to aggregate multi-scale feature maps from different ResNet blocks [35]. By extending RPN-FPN module [36] to 3D, Voxel-FPN [37] uses feature pyramid to aggregate voxel features of different voxelization resolutions. We also utilize the multi-scale feature modeling strategy, but are to balance the accuracy and efficiency of the voxel branch for point-voxel convolution, which has not been investigated before.

### 2.3. Attention Mechanism

Attention is originally a physiological mechanism that describes the phenomenon that humans' perception system could focus on the object of interest while suppressing the background [38]. Inspired by it, deep learning researchers attempt to exploit it to analyze networks' focus [39, 40] or enforce neural networks to focus on more important features [41, 42].

Attention is also widely adopted to model the relationship between two instances, e.g., generating the most relevant sentences for images in the task of image caption [43] or searching the most relevant sentences between two different languages in the task of machine translation [44]. By projecting the query instance into the same high-dimensional space as the target, relevant spatial regions of the query will be highlighted to guide the desired inference. We also aim to model the relationship. Differently, our inferred relevance is used for the fusion of features extracted from the voxel branch and point branch during point-voxel convolution.

## 3. Method

In this section, we will first review the architecture of PVConv, analyze the factors that may limit its performance and then introduce the overview of our solution, i.e., pyramid point-voxel convolution (PyraPVConv). After that, we describe the two main components of PyraPVConv: the voxel pyramid module and the sharable attention module.

### 3.1. Review of PVConv [20]

Methodology of PVConv Given an unordered point set **P**={(*p*_*k*_, *f*_*k*_)} with {*p*_*k*_} denoting the point coordinates and {*f*_*k*_} as the point features, PVConv adopts an isolated *point branch* to extract individual point features using MLPs similar to PointNet. Apart from that, another *voxel branch* in PVConv is utilized to facilitate efficient and powerful neighbourhood feature aggregation. Particularly, the feeded voxels to the voxel branch are generated by first normalizing the point coordinates and then conducting voxelization to transform the normalized point cloud $\left\{\left(\hat{p_{k}},f_{k}\right)\right\}$ into a volume **V** by averaging all features {*f*_*k*_} whose normalized coordinates $\left\{\hat{p_{k}}\right\}$ fall into that voxel grid.

The article "PyraPVConv: Efficient 3D Point Cloud Perception with Pyramid Voxel Convolution and Sharable Attention" was published in 2022. Journal: Comput Intell Neurosci.

Finally, the two-branch features are linearly fused, i.e., the voxel features are devoxelized to the point cloud domain using trilinear interpolation, and then added with point features.

Discussion on PVConv As mentioned in PVConv, the MLPs in the *point branch* can already output discriminative features for each point. Therefore, the main contribution of PVConv is to leverage *the voxel branch* for neighborhood feature aggregation.

However, perhaps focusing too much on the efficiency factor, PVConv is *conservative* in utilizing the *voxel branch*, e.g., very limited volume resolutions and 3D convolution layers are adopted. Indeed, 3D convolutions that are derived from mature 2D convolution techniques are powerful, and have a good tradeoff between accuracy and efficiency. Furthermore, simple trilinear interpolation would lead to information loss of those voxel features that are not sufficient originally.

### 3.2. Overview of PyraPVConv

To resolve the above issues of PVConv, we propose a novel PyraPVConv block with two key structural modifications: a voxel pyramid module for the voxel branch and a sharable attention module for feature fusion. Similar as in PVConv, the point branch of PyraPVConv extracts individual point features. At the same time, the voxel branch of PyraPVConv adopts the voxel pyramid module to extract more powerful voxel features in pyramid. Then, the shareable attention module fuses point features and voxel features in pyramid nonlinearly. Please refer to Figure 1 for a demonstration.

### 3.3. Voxel Pyramid Module

To extract sufficient voxel features without bringing too much additional computational overhead, we propose a voxel pyramid module to capture multiscale features in different pyramid levels, inspired by [36]. Please refer to Figure 2 for a demonstration.

Volume Generation Given the normalized point cloud $\left\{\left(\hat{p_{k}},f_{k}\right)\right\}$ as in PVConv, we generate a volume by averaging all features {*f*_*k*_} whose coordinates $\left\{\hat{p_{k}}\right\}$ fall into that voxel grid via the following equation:

(1) $$\begin{array}{c} V_{r}\left(u,v,w\right)=\frac{1}{N_{r,u,v,w}}\sum_{k=1}^{N}I\left(\left\lfloor x_{k}\times r\right\rfloor =u,\left\lfloor y_{k}\times r\right\rfloor =v,\left\lfloor z_{k}\times r\right\rfloor =w\right)\times f_{k,c}, \end{array}$$

where *r* denotes the volume resolution, *N*_*r*,*u*,*v*,*w*_ denotes the number of points falling in the voxel grid (*u*, *v*, *w*) of volume **V**_*r*_, *f*_*k*,*c*_ denotes the *c*^th^ channel corresponding to ${\hat{p}}_{k}$, and *𝕀*() is a binary indicator function.

The article "PyraPVConv: Efficient 3D Point Cloud Perception with Pyramid Voxel Convolution and Sharable Attention" was published in 2022. Journal: Comput Intell Neurosci.

Bottom-up Feature Extraction Given **V**_*r*_, we feed it to the same 3D voxel convolution networks as in PVConv, i.e., two groups of conv3d, batch normalization and activation layers, to obtain 3D voxel feature *f*_*r*_^**V**^,

(2) $$\begin{array}{c} f_{r}^{V}={\text{Conv}3\text{D}}_{1}\left(V_{r}\right). \end{array}$$

Unlike PVConv that adopts a conservative strategy in the voxel branch, we suggest making full use of the features in volume **V**_*r*_. Considering the efficiency, we conduct an average pooling operation with a scaling rate of 1/2 to *f*_*r*_^**V**^, and then feed it another 3D voxel convolution networks,

(3) $$\begin{array}{c} f_{r/2}^{V}={\text{Conv}3\text{D}}_{2}\left(\text{MaxPool}\left(f\left(\begin{array}{c} V\\ r \end{array}\right)\right)\right.. \end{array}$$

We apply the same operations iteratively to obtain multi-scale 3D voxel features. In this paper, we adopt three-scale features *f*_*r*_^**V**^, *f*_*r*/2_^**V**^, and *f*_*r*/4_^**V**^.

To-down Feature Aggregation Given each 3D voxel feature, we enhance it by aggregating with the feature of a higher pyramid level (if has) that is spatially coarser but semantically strong. It is implemented by applying an upsampling operation followed with addition,

(4) $$\begin{array}{c} {\hat{f}}_{r/4}^{V}=f_{r/4}^{V},\\ {\hat{f}}_{r/2}^{V}=\text{UpPool}\left({\hat{f}}_{r/4}^{V}\right)+f_{r/2}^{V},\\ {\hat{f}}_{r}^{V}=\text{UpPool}\left({\hat{f}}_{r/2}^{V}\right)+f_{r}^{V}. \end{array}$$

Therefore, we obtain three semantic enhanced voxel features: ${\hat{f}}_{r}^{V}$, ${\hat{f}}_{r/2}^{V}$, and ${\hat{f}}_{r/4}^{V}$.

### 3.4. Sharable Attention Module

With enhanced voxel features ${\hat{f}}_{r}^{V}$, ${\hat{f}}_{r/2}^{V}$, ${\hat{f}}_{r/4}^{V}$ and point features {*f*_*k*_} as inputs, we fuse them via using the attention mechanism. Since voxel features in different pyramid levels contain discriminative but complementary information, we apply attentive fusion of them with point features separately. It is implemented by converting the voxel features into the same feature space as point features, and then summarize them. See Figure 3 for a demonstration. In the following, we will describe the attention method taking ${\hat{f}}_{r}^{V}$ as an example.

The article "PyraPVConv: Efficient 3D Point Cloud Perception with Pyramid Voxel Convolution and Sharable Attention" was published in 2022. Journal: Comput Intell Neurosci.

Attentive Fusion for a Pyramid Level Instead of fusing all voxel features, we only consider eight neighboring voxel features $\left\{{\hat{f}}_{r}^{V}\left(k,m\right)\right\}$ with *m*=1,2,…, 8 for each point $\left\{\left(\hat{p_{k}},f_{k}\right)\right\}$ following PVConv, considering the tradeoff between efficiency and performance. Specifically, we adopt a similar attention process to that in [45] with three key steps. First, we project point feature *f*_*k*_ and its eight neighboring voxel features $\left\{{\hat{f}}_{r}^{V}\left(k,m\right)\right\}$ into the same feature space using two networks *Q*_*r*_ and *K*_*r*_. Second, we calculate the relevant scores between eight voxel features and that point feature by conducting dot product of their flattened features. Note that, we also adopt the Sigmoid operation to enforce the relevant scores to be between 0 and 1.

(5) $$\begin{array}{c} \text{Rel}\left(f_{k},{\hat{f}}_{r}^{V}\left(k,m\right)\right)=\text{Sigmoid}\left(Q_{r}\left(f_{k}\right)\times K_{r}\left({\hat{f}}_{r}^{V}\left(k,m\right)\right)\right). \end{array}$$

Finally, we convert the voxel features $\left\{{\hat{f}}_{r}^{V}\left(k,m\right)\right\}$ into a summable space with point features using the network *H*_*r*_, and then aggregate them weighted with the relevant scores $\text{Rel}\left(f_{k},{\hat{f}}_{r}^{V}\left(k,m\right)\right)$.

(6) $$\begin{array}{c} f_{k}^{\prime }=f_{k}+\sum_{m}H_{r}\left({\hat{f}}_{r}^{V}\left(k,m\right)\right)\text{Rel}\left(f_{k},{\hat{f}}_{r}^{V}\left(k,m\right)\right). \end{array}$$

Multiple Pyramid Fusion with Sharable Attention For voxel features in all three pyramid levels, we apply the above attentive fusion method, and then summarize them together.

(7) $$\begin{array}{c} {\hat{f}}_{k}^{\prime }=f_{k}+\sum_{r}\sum_{m}H_{r}\left({\hat{f}}_{r}^{V}\left(k,m\right)\right)\text{Rel}\left(f_{k},{\hat{f}}_{r}^{V}\left(k,m\right)\right). \end{array}$$

Therefore, ${\hat{f}}_{k}^{\prime }$ is the final fused feature that contains both point and voxel features. Particularly, since the inputs for networks *Q*_*t*_ with *t*=*r*, *r*/2, *r*/4 are exactly the same, we simply use one network *Q* and share it with all three pyramid levels for efficiency purpose.

## 4. Experimental Results

To validate the effectiveness and efficiency of PyraPVConv, we extensively evaluate the performance of PyraPVCNN, which is constructed by stacking multiple PyraPVConv blocks, on three different tasks, i.e., indoor scene segmentation, object part segmentation and 3D object detection.

### 4.1. Implementations

For PyraPVCNN, we replace all the PVConv blocks in PVCNN with PyraPVConv and use the same decoding layer. We implement PyraPVCNN and reproduce all the evaluated networks with PyTorch for fair comparisons, and report the latency and memory consumption at test time on a workstation with an Intel Xeon E5-2678 CPU@2.5 Hz and 64 GB of memory using a single RTX 2080Ti GPU.

The article "PyraPVConv: Efficient 3D Point Cloud Perception with Pyramid Voxel Convolution and Sharable Attention" was published in 2022. Journal: Comput Intell Neurosci.

### 4.2. Indoor Scene Segmentation

Setups We conduct semantic segmentation experiments on the large-scale Stanford 3D semantic parsing dataset (S3DIS) [47, 48]. S3DIS is scanned across 271 rooms in 6 areas with a Matterport camera (combined with 3 structured light sensors at different intervals), and then each point in the scanned point cloud is annotated with a semantic label (e.g., a total of 13 objects such as chairs, tables, floors, walls, etc.). We adopt the same data processing procedure as PVCNN [20]. We train the models on regions 1, 2, 3, 4, and 6 and test them on region 5 to evaluate the mean intersection-over-union (mIoU) and the mean class-wise accuracy (mAcc), with both metrics measured as percentages.

Models Six state-of-the-art methods are adopted as baselines: PointNet [20], PointNet++ [18], DGCNN [25], PointCNN [46], PVCNN [20] and RandLA-Net [27]. Since our focus is on the efficiency of deep networks, similar as in PVCNN, we also evaluate the narrower versions of PVCNN and PyraPVCNN by reducing the number of feature channels from that of the original version (denoted as 1 × *C*) to 12.5% (denoted as 0.125 × *C*), 25% (denoted as 0.25 × *C*) and 50% (denoted as 0.5 × *C*).Comparison Results The results reported in Table 1 show that Ours (0.125 × *C*) performs better than two state-of-the-art point-based methods: PointNet [11] and DGCNN [25] and voxel-based methods: PVCNN (0.25 × *C*) [20], and is comparable to the state-of-the-art RandLA-Net [27], but with less latency and GPU memory consumption. In addition, the performance of Ours (1 × *C*) is nearly 10% higher than that of DGCNN [25], but the latency is reduced by 20%, and GPU memory consumption is reduced by 1.6 times. In particular, Ours (0.25 × *C*) outperforms the full version of PVCNN, but the latency and GPU memory consumption are much less. Please refer to Figure 4 to see an illustrative demonstration of the tradeoff between accuracy (mIoU) and the incurred overhead (the number of parameters, latency and GPU memory consumption).

We also visualize the segmentation results in Figure 5. It could be seen that Ours (0.25 × *C*) can better utilize neighborhood information to improve the prediction of point labels, compared with PVCNN.

Ablation Studies To validate the importance of the two key modules of PyraPVConv: voxel pyramid module and the sharable attention module, we report the results of ablation studies using two narrow versions of the PyraPVCNN (i.e., 0.25 × *C* and 0.5 × *C*) in Table 2. It could be seen that the performance will drop, if we delete any one of them. In particular, the voxel pyramid module has a slightly larger impact on the performance.

The article "PyraPVConv: Efficient 3D Point Cloud Perception with Pyramid Voxel Convolution and Sharable Attention" was published in 2022. Journal: Comput Intell Neurosci.

### 4.3. Object Part Segmentation

Setups We choose the ShapeNet Parts dataset [49] to conduct the experiment of object part segmentation. ShapeNet Parts is a collection of 16681 point clouds selected from 16 categories of the ShapeNetCore, and is manually annotated with a total of 50 parts. Following [46], we train the models on 14006 point clouds, evaluate the part-averaged IoU for each of the remaining 2874 point clouds, and then average them as the final metric, i.e., mIoU (%).

Models We choose point-based models: PointNet [11], PointNet++ [18], and DGCNN [25] and the voxel-based model: 3D-UNet [50], and PVCNN [20] as baselines.

Comparison Results As shown in Table 3, Ours (0.25 × *C*) performs much better while the latency is 36 times lower and the GPU memory consumption is 11.7% lower than that of 3D-UNet. Moreover, it is superior to the most advanced point-based methods such as PointNet [11], PointNet++ [18] and DGCNN [25] in all aspects. In particular, we would like to emphasize that Ours (0.5 × *C*) outperforms PVCNN [20], and Ours (1 × *C*) outperforms PointCNN [46] with only about 58% latency and GPU memory consumption. Please refer to the visualization results in Figure 6 for intuitive comparisons.

### 4.4. 3D Object Detection

Setups We conduct 3D object detection experiments on the large outdoor dataset KITTI [51]. KITTI provides 7481 training and verification samples for objects such as cars, pedestrians, and cyclists, of which 3711 samples are used for training and the remaining 3769 samples are for verification. We evaluate all models 20 times and report the average 3D average accuracy (AP) measured as percentages.

Models We build multiple Frustum Networks [29] with PointNet [11], PointNet++ [18], PVCNN [20], a narrow version of PyraPVCNN (0.25 × *C*) as backbones.

Comparison Results As shown in Table 4, the Frustum Network with PyraPVCNN (0.25 × *C*) (denoted as F-PyraPVCNN) as backbone outperforms than all three other Frustum Networks with PointNet [11], PointNet++ [18] and PVCNN [20] as backbones (denoted as F-PointNet, F-PointNet++ and F-PVCNN), but with much less latency and GPU memory consumption. In particular, F-PyraPVCNN (0.25 × *C*) improves the detection rate of pedestrian by 4% compared with the F-PVCNN, and 7.5% compared with the F-PointNet, validating the usefulness of PyraPVCNN in 3D detection tasks.

## 5. Conclusion

In this paper, we have presented a novel PyraPVConv block with the aim of efficient 3D point cloud perception. The key idea is to utilize voxel pyramid to make full use of voxel information and then adopt the attention mechanism for better point-voxel feature fusion. Extensive experiments validate the superiority of PyraPVConv. We hope that PyraPVConv can act as an important part of various deep networks for 3D point cloud perception. In the future, we plan to utilize the technique of neural architecture search for designing more efficient network architectures.

The article "PyraPVConv: Efficient 3D Point Cloud Perception with Pyramid Voxel Convolution and Sharable Attention" was published in 2022. Journal: Comput Intell Neurosci.

## Figures and Tables

**Figure 1:** The architecture of PyraPVConv, with a point branch extracting single point features, and a voxel branch aggregating neighborhood information via a voxel pyramid module and an sharable attention mechanism.

**Figure 2:** Demonstration of the bottom-up feature extraction and top-down feature aggregation in the voxel pyramid module.

**Figure 3:** Demonstration of the sharable attention module.

**Figure 4:** The tradeoff between accuracy and the number of parameters, measured latency, and GPU memory consumption for PyraPVCNN and the state-of-the-art baselines on S3DIS. (a) Parameters (M), (b) Latency (ms), (c) GPU memory (GB).

**Figure 5:** Visualization of the semantic segmentation results on the S3DIS dataset.

**Figure 6:** Visualization of object part segmentation results on the ShapeNet Parts dataset.

**Table 1:** Indoor scene segmentation results on the S3DIS dataset. Note that the input data of PointCNN [46] include 16 × 2048 points, while the data of the other methods include 8 × 4096 points.

	mAcc	mIoU	Latency (ms)	GPU mem. (GB)	#Param.
PointNet	82.54	42.97	16.1	1.50	3.53 M
PVCNN (0.125 × *C*)	82.60	46.94	7.6	0.46	43.16 K
DGCNN	83.64	47.94	79.0	4.50	987.00 K
PVCNN (0.25 × *C*)	84.52	51.96	11.4	0.76	166.21 K
**Ours** (0.125 × *C*)	84.88	**52.16**	10.3	0.59	143.19 K

PVCNN (0.5 × *C*)	85.88	54.73	17.5	0.97	650.35 K
PVCNN	86.25	55.54	35.9	1.92	2.57 M
**Ours** (0.25 × *C*)	86.49	**55.86**	21.6	1.04	693.72 K

**Ours**(0.5 × *C*)	86.93	57.02	41.3	1.84	1.82 M
PointCNN	85.91	57.26	282.3	4.60	5.86 M
RandLA-Net	85.10	**58.60**	911.1	2.57	4.76 M
**Ours**(1 × *C*)	**86.96**	57.98	71.2	2.52	3.13 M

**Table 2:** The indoor scene segmentation performance on the S3DIS dataset with ablating the voxel pyramid module (VPM.) and the sharable attention module (ASM.).

Channel	Metric	Ours	W/o VPM.	W/o ASM.
0.25 × *C*	mIoU	**55.86**	53.01	53.87
	mAcc	**86.49**	84.91	85.56
0.5 × *C*	mIoU	**57.02**	55.07	55.68
	mAcc	**86.93**	85.67	86.31

**Table 3:** Object part segmentation results on the ShapeNet Parts dataset.

	Input data	Convolution	mIoU	Latency (ms)	GPU mem. (GB)
PointNet	Points (8 × 4096)	None	83.70	16.0	1.5
3D-UNet	Voxels (8 × 963)	Voxel-based	84.60	480.0	17.6
PointNet++	Points (8 × 4096)	Point-based	84.70	55.6	4.0
DGCNN	Points (8 × 4096)	Point-based	84.70	61.8	4.8
PVCNN (0.25 × C)	Points (8 × 4096)	Voxel-based	84.72	10.1	1.2
**Ours**(0.25 × C)	Points (8 × 4096)	Voxel-based	**85.12**	13.2	1.5

PVCNN (0.5 × C)	Points (8 × 4096)	Voxel-based	85.38	17.5	1.8
PVCNN	Points (8 × 4096)	Voxel-based	85.70	35.2	3.1
**Ours** (0.5 × C)	Points (8 × 4096)	Voxel-based	**85.97**	29.7	2.4

PointCNN	Points (16 × 2048)	Point-based	86.10	95.6	5.1
**Ours**(1 × *C*)	Points (8 × 4096)	Voxel-based	**86.82**	56.7	3.2

The article "PyraPVConv: Efficient 3D Point Cloud Perception with Pyramid Voxel Convolution and Sharable Attention" was published in 2022. Journal: Comput Intell Neurosci.

**Table 4:** 3D object detection results of the Frustum Networks [29] on the validation set of KITTI with different backbones.

Backbone	Efficiency		Car			Pedestrian			Cyclist		
	Latency (ms)	GPU mem. (GB)	Easy	Mod.	Hard	Easy	Mod.	Hard	Easy	Mod.	Hard
PointNet	29.1	1.5	83.26	69.28	62.56	65.08	55.85	49.28	74.54	55.95	52.65
PointNet++	101.2	2.5	83.76	70.92	63.65	70.00	61.32	53.59	77.15	56.49	53.37
PVCNN	51.9	1.9	84.22	71.11	**63.66**	69.16	60.28	52.52	78.67	57.79	54.16
Ours (0.25 × *C*)	**39.6**	**1.4**	**85.42**	**71.24**	63.09	**71.80**	**64.67**	**56.87**	**79.32**	**58.57**	**55.01**

## Data Availability

All datasets used in this paper are publicly available.
